The article "Classification of Lactate Level Using Resting-State EEG Measurements" was retracted in 2023. Reasons: signs of a paper mill; suspected computer-generated content; unreliable results or conclusions; lack of ethics approval or compliance.

# Classification of Lactate Level Using Resting-State EEG Measurements

**DOI:** 10.1155/2021/6662074

**Published:** 2021-02-08

**Authors:** Saad Abdulazeez Shaban, Osman Nuri Ucan, Adil Deniz Duru

**Affiliations:** ^1^Computer Science Department, College of Education for Pure Sciences, Diyala University, Diyala 32001, Iraq; ^2^Electrical and Computer Engineering, School of Engineering and Natural Sciences, Altınbaş University, Istanbul 34217, Turkey; ^3^Engineering Faculty, Electrical and Electronics Department, Istanbul University, 34850 Avcilar, Istanbul, Turkey; ^4^Neuroscience and Psychology Research in Sports Lab, Faculty of Sport Science, Marmara University, 34668 Istanbul, Turkey

## Abstract

The electroencephalography (EEG) signals have been used widely for studying the brain neural information dynamics and behaviors along with the developing impact of using the machine and deep learning techniques. This work proposes a system based on the fast Fourier transform (FFT) as a feature extraction method for the classification of human brain resting-state electroencephalography (EEG) recorded signals. In the proposed system, the FFT method is applied on the resting-state EEG recordings and the corresponding band powers were calculated. The extracted relative power features are supplied to the classification methods (classifiers) as an input for the classification purpose as a measure of human tiredness through predicting lactate enzyme level, high or low. To validate the suggested method, we used an EEG dataset which has been recorded from a group of elite-level athletes consisting of two classes: not tired, the EEG signals were recorded during the resting-state task before performing acute exercise and tired, the EEG signals were recorded in the resting-state after performing an acute exercise. The performance of three different classifiers was evaluated with two performance measures, accuracy and precision values. The accuracy was achieved above 98% by the K-nearest neighbor (KNN) classifier. The findings of this study indicated that the feature extraction scheme has the ability to classify the analyzed EEG signals accurately and predict the level of lactate enzyme high or low. Many studying fields, like the Internet of Things (IoT) and the brain computer interface (BCI), can utilize the findings of the proposed system in many crucial decision-making applications.

## 1. Introduction

Electroencephalography is the brain neural signals which reflect the brain's electrical potentials and are mainly used for studying brain neural information dynamics processing and employed to diagnose brain disturbances [1]. Normally, those signals are time series signals [2] recorded by means of a specialized skull helmet which contains multiple electrodes distributed and attached to a specific position on the scalp, either in a wet or dry manner [3]. The data acquired from the recording of such signals are in a very large amount, and that is why they should be analyzed by specialized methods, rather than conventional visual ways [4]. Among those methods, data classification using machine learning techniques can play a vital role in analyzing and investigating EEG signals and exploitation results in different applications like diagnosing human mental diseases [5], predicting emotional states, decision discovery for patient rehabilitation devices, or assistive technology for interactive input devices like gaming controllers and wheelchairs drivers [6]. Many of the previous studies were investigating different brain activity by means of magnetic resonance imaging (MRI) that measures anatomical images noninvasively. Resting-state functional MRI activity is shown to differ between before and after performing aerobic exercise [7]. A recent study investigates the impact of a single acute exercise session on the brain's functional connectivity and showed an obvious increase in the functional connectivity of sensorimotor brain networks that could be clearly assessed using functional MRI [8]. Even though the MR imaging shows high spatial resolution, but because of the blood oxygenated level dependency attributes (BOLD), it shows a limited temporal resolution of the measured signals. Using the electroencephalography signals as a measure of electrophysiological brain activity produces enhancement in temporal resolution to a range of milliseconds [9]. The use of EEG as a technique of analyzing in the field of psychology has been applied for a long time in many studies, but it was not that common in the field of exercises and sports until recent times. A study investigated the impact of severe physical short-term exercise and long-term workout training on the EEG resting-state alpha frequency (iAPF) of the individual shows that frequency has increased after performing intense exercise [10], while another study shows an increment in the power of the frontal area observed in the EEG signals after performing acute cycling exercises [11]. The high-intense running was found to have an effect on both EEG and the mood of the exerciser [12]. Brain activation during aerobic exercises was found to be increased, i.e., the EEG beta frequency band power is increased and the alpha frequency band is decreased during performing moderate-intensity short-time cycle ergometer exercise, then returning to the power baseline after finishing [13].

The article "Classification of Lactate Level Using Resting-State EEG Measurements" was retracted in 2023. Reasons: signs of a paper mill; suspected computer-generated content; unreliable results or conclusions; lack of ethics approval or compliance.

One of the emerging aspects in this field is predicting the lactate dehydrogenase enzyme levels, whether being high or low, in the human blood by classifying the collected resting-state EEG data [14] from a subject along with measuring lactate levels in the blood. The idea behind that is to study whether lactate levels in the human blood could be predicted of being increased or decreased affected by performing an acute exercise, as it was reported that the blood lactate level would reach its peak after maximal treadmill running exercise was made for a short period [15], meanwhile collecting EEG data before and after exercise and mark them as class 1 (before exercise or lactate-level-low) and class 2 (after exercise or lactate-level-high). This study is aimed at examining this idea by suggesting a classification system that should discriminate two states of lactate level using EEG signals having different frequency bands recorded from a group of healthy athlete subjects of the elite level, before and after performing a single bout of acute exercise. As EEG signals have different features that could be extracted using a variety of methods [16], we should dominate the best discriminant feature that gives us the best classification score in terms of accuracy. Among different features, the band power features which represent the energy (power) of EEG signals were chosen to represent a discriminant criterion and are computed by means of power spectral density of each EEG signal frequency band for a given channel. Frequency band power is regarded as a gold standard feature to be applied in applications like brain computer interface (BCI) by many studies [6, 17]. Band power features are calculated to evaluate the brain's activity changes over a given time window (typically of a few seconds) encountered by performing an acute exercise session. Then, the extracted feature data is arranged in a vector, manipulated and modified using preprocessing techniques to clean data from artifacts and enhance the model performance. These features are analyzed along with the relation to blood lactate levels before and after performing exercises. To the best of the author knowledge, until now, no one study in the literature is related to the assessment of classification performance using power spectral density- (PSD-) based feature extraction machine learning classifiers when applied to the fatigue problem after acute exercise. Compared with several studies, experimental results clarify that the suggested system could enhance the detection rate.  Figure 1 shows the schematics of the proposed system.

## 2. Materials and Methods

### 2.1. Operational Tasks

In this study, the employed dataset that includes the resting-state EEG signals from [9], has been used. The proposed system in our study consists of two main parts: one involves feeding lactate enzyme level test measurements, and the other involves input the EEG signal recordings and manipulating them. EEG data was recorded from a volunteers' group of elite level athletes (no.of subjects = 10), and all are representing members of official karate team. These subjects had performed the blood lactate level test before doing the exercise, and the results were allocated to represent low-level lactate (not tired) class. Initial lactate measurements were found to be at the baseline value of around 2 millimoles/litre. In the first step, subjects were sitting in a calm fashion with eyes closing (EC) condition and asked to stay as-calm-as possible and thinking about nothing for 3 minutes. Meanwhile, the EEG signals are being collected from subjects with a sampling rate of 1000 Hz using BrainAmp ExG amplifier from 16 channels (Fz, Fp1, Fp2, F3, F4, Cz, C3, C4, T7, T8, Pz, P3, P4, Oz, O1, and O2) with dry electrode caps.  Figure 2 shows the distribution of 16 electrodes over the brain scalp.

The article "Classification of Lactate Level Using Resting-State EEG Measurements" was retracted in 2023. Reasons: signs of a paper mill; suspected computer-generated content; unreliable results or conclusions; lack of ethics approval or compliance.

The next step in this phase requires each subject to separately perform an acute exercise of a short-time shuttle run with 20 meters for each shuttle. This running protocol is an incrementally progressive test that is used to predict personal physical sensations experienced during exercises like maximum oxygen consumption, increased heart rate, muscle fatigue, and increased sweating. It consists of 20 m running that requires increasing running pace while time decreases as levels proceed with a beep stimulus between levels.

While performing the exercise, the performance is monitored using rated perceived exertion (RPE) scale. RPE is a scale for measuring physical activity intensity by asking the activist about how he feels his body is working without interrupting the exercise. The exercise ended when each subject reports a 16 RPE level according to the Borg rating of perceived exertion [18].

The next experimental phase starts, after a short resting period of one minute, by measuring blood lactate levels for each subject, and it was found at a high level of around 16 millimoles/litre. Then, the lactate test is repeated 4 times with 2 minutes between them, and each test result found to be at the same high levels with no drop to baseline within the EEG data measurement phase. Then, the EEG data measuring was repeated with EC condition for 3 minutes and assigned to be a high-level lactate (tired) class. Both datasets of measured EEG signal, pre, and postexercise contain artifacts generated by some muscular movement, eye blinking, and heartbeats that can contaminate the quality of EEG data [19], and that is why the data has been cleaned from noises by removing epochs that have an absolute amplitude greater than 100 *μ*V by using band-pass filtering technique.  Figure 3 shows epochs of 1 second EEG signal of one subject recorded from 16 channels before and after performing the exercise.

The article "Classification of Lactate Level Using Resting-State EEG Measurements" was retracted in 2023. Reasons: signs of a paper mill; suspected computer-generated content; unreliable results or conclusions; lack of ethics approval or compliance.

### 2.2. Feature Extraction

The EEG signals are nonstationary time-series signals, and once the raw version of EEG data was recorded then passed the preprocessing step, the next step is to get related attributes through the feature extraction process. To get the better distinguishing feature from EEG signals, we have applied the fast Fourier transform (FFT) method to provide frequency representation of the signals, which helps to measure the power spectrum of data for each frequency band, delta (0-4 Hz), theta (4-8), alpha (8-13), beta (13-30), and gamma (30-45), within a time window or epoch. For the frequency spectral analysis, the nonstationarity can be tolerated and the EEG signal assumed stationary for the epoch period. Fast Fourier transform (FFT) is a signal processing method which is used to transform the signal from its time domain to the equivalent frequency domain representation by dividing the signal function into a continuous frequency band known as frequency spectrum [20]. If *F*(*k*) is the fast Fourier transform of a function *f*(*z*), then it is defined by using equation (1) as follows:

(1) $$\begin{array}{c} F\left(k\right)=\underset{z\text{ even}}{\sum }f\left(z\right)w_{Z}^{kz}+\underset{z\text{ odd}}{\sum }f\left(z\right)w_{Z}^{kz}, \end{array}$$

for *k* = 0, 1, .⋯., *Z* − 1, where *F*(*k*) is the Fourier coefficient of *f*(*z*), which is assumed to have a complex value, *z* even and *z* odd correspond to the EEG samples of *f*(*z*), which were even and odd numbered, respectively. *w* = exp (−2*zj*/*Z*), where *z* is equal to 3.14, and *j* is the imaginary part.

### 2.3. Classification

The process of EEG data formatting and performing frequency band power calculation is done by a self-developed MATLAB routine, and the resulting data, pre, and postexercise are then combined and formed a single bulk dataset of size 7759 rows and 80 columns and fed to a set of classification algorithms (classifiers) with 80 features and two class labels, “1” is representing lactate-level-low before exercise, and “2” is representing lactate-level-high after exercise. Among those applied classifiers, the KNN, decision tree (DT), and logistic regression (LR) have reported scoring better than others, like the linear discriminant analysis (LDA) classifier and support vector machine (SVM) classifier; thus, only the highest-scoring classifiers have been listed in Results.

The article "Classification of Lactate Level Using Resting-State EEG Measurements" was retracted in 2023. Reasons: signs of a paper mill; suspected computer-generated content; unreliable results or conclusions; lack of ethics approval or compliance.

#### 2.3.1. Decision Tree

A decision tree is a machine learning model in which each nonleaf node denotes a test on a feature, each branch node represents an outcome of the test, and each terminal node holds a class label. The root node is the topmost node. Assume an X tuple with an unknown class label, the feature values of X are tested against the tree with path traced along from the root node to a leaf node, which represents the class prediction for the given tuple [21]. Each decision tree employs an attribute selection method that specifies a procedure for choosing the best attribute that discriminates the tuple depending on the class. This procedure uses attribute selection measure as a metric function to evaluate split for feature selection such as the information gain and the Gini index. Some attribute selection measures impose the tree to become binary like the Gini index; others like information gain are not. Gini index measures the impurity of data from a set of training tuples, as in equation (2).

(2) $$\begin{array}{c} \text{Gini}\left(\text{data}\right)=1-\overset{k}{\underset{i=1}{\sum }}{Pi}^{2}, \end{array}$$

where *Pi* represents the probability that a tuple in data belongs to a specific class, say *Ci*. Information gain is an attribute selection measure that tries to find the attribute which has the highest information gain that minimizes the required information to classify tuple and is defined by equation (3).

(3) $$\begin{array}{c} \text{Inf}\left(\text{data}\right)=-\overset{k}{\underset{i=1}{\sum }}Pi\log_{2}\left(Pi\right), \end{array}$$

where *Pi* is the probability that a tuple in data belongs to a specific class *Ci*.

#### 2.3.2. K-Nearest Neighbor

The K-nearest neighbor (KNN) classifiers learn by comparing a given test vector with similar training vectors (SRs). The training vectors are described by number of *n* attributes. When given an unknown vector, a K-nearest neighbor classifier seeks the pattern field for the k training vectors (nearest neighbors) that are closest to the unknown vector. The “closeness” is defined in terms of a distance, such as Manhattan distance, which defines distance d between *x*1 and *x*2 vectors, as in equation (4):

(4) $$\begin{array}{c} d\left(j,l\right)=\left|xj1-xl1\right|+\left|xj2-xl2\right|+\left|xj3-xl3\right|. \end{array}$$

Then, the probability is used as a measure to assign the input *x* to the most probable class (nearest one), as in equation (5):

(5) $$\begin{array}{c} P\left(y=j\;|\;X=x\right)=\frac{1}{K}-\underset{i∊B}{\sum }L\left(y^{\left(i\right)}=j\right), \end{array}$$

where *B* represents the set of K neighbors of the training vector which are nearest to input *x*, and *L*(*x*) represents indicator that acts as a function which sets to 1 if the input *x* is true and set to 0 if not.

The article "Classification of Lactate Level Using Resting-State EEG Measurements" was retracted in 2023. Reasons: signs of a paper mill; suspected computer-generated content; unreliable results or conclusions; lack of ethics approval or compliance.

#### 2.3.3. Logistic Regression

Logistic regression is a popular model for solving classification problems, and the term “Logistic” comes from the underlying Logit function used in this model for classification, the natural logarithm of odds ratio [22]. Logistic regression estimates as probability the impacts of independent variables on the outcome variables. Simple logistic model is shown in equation (5).

(6) $$\begin{array}{c} \text{Logit}\left(y\right)=\text{naturallog}\left(\text{odds}\right)=\ln\left(\frac{y}{1-y}\right), \end{array}$$

where the logit(*y*) is representing the probabilities from 0 to 1.

The technology used for classification was the Classification Learner applications available in the MATLAB R2018a software.

To validate entire input data, we used the technique of K-fold cross-validation, which splits data into K folds (parts). Among these K folds, K-1 folds are used to train proposed model and the remaining fold is used for testing purpose. The procedure is replicated for K times until all subsets are validated; then, all the results are averaged for final accuracy prediction [23].

## 3. Results

The extraction of EEG band power feature yields a significant enhancement in the classifier's accuracy scores, especially for KNN, decision tree and logistic regression classifiers. The main finding of our study is proving the ability to clearly predict human blood lactate levels using resting-state EEG signals when applying suitable techniques, power spectral density in our case. The classification score versus applied method results are listed in the Table 1. To the best of the authors' knowledge, there is no study in the literature related to the classification performance measure using FFT and machine learning classifiers, investigating the fatigue problem after acute exercise.

Another measure is to calculate the specificity and sensitivity of the classifier. Sensitivity is also referred to as the rate of true positive recognition (i.e., the proportion of the first-class belonging tuples that are correctly identified); on the other hand, specificity represents the rate of true negative recognition (i.e., the proportion of the second-class belonging tuples that are correctly identified) [24]. These two measures are defined as follows in equations (6) and (7), respectively:

(7) $$\begin{array}{c} \text{Sensitivity}=\frac{\text{TP}}{\text{TP}+\text{FP}}, \end{array}$$

(8) $$\begin{array}{c} \text{Specificity}=\frac{\text{TN}}{\text{TN}+\text{FN}}, \end{array}$$

where TP represents the positive tuples of data that were correctly classified by the model, whereas FP represents the positive tuples that were falsely classified. On the other hand, TN represents the negative tuples of data that were correctly classified by the model. In contrast, FN represents the negative tuples that were falsely classified by the model.  Table 2 shows those measures for each of the applied classification models. Thus, we note that the KNN and decision tree classifiers have a high accuracy along with high sensitivity and specificity which indicates their ability to correctly classify both the positive and negative tuples, which are in contrast to the logistic regression classifier that showed a moderate sensitivity and specificity scores meaning that it can recognize positive and negative tuples at a lower rate.

The article "Classification of Lactate Level Using Resting-State EEG Measurements" was retracted in 2023. Reasons: signs of a paper mill; suspected computer-generated content; unreliable results or conclusions; lack of ethics approval or compliance.

Furthermore, classifiers show the following precision values, which represent percentage of instances labelled as positive and are actually such, for both classes, lactate-level-low and lactate-level-high denoting pre-exercise (not tired) and post-exercise (tired) tiredness recognition, respectively, for different classifiers as in Table 3a, b, and c as follows:

## 4. Discussion

In the present study, we had investigated the ability to predict whether the lactate level is low or high in the human body using EEG signals of subjects after performing an acute exercise. The subjects were athletes of the elite level from the national team of Turkey. The achieved results indicate that predicting blood lactate levels, high or low, using electroencephalogram brain data can be done accurately in terms of classification scores when implemented for healthy athlete who endures a single bout of acute exercises. The discrimination ability is driven by the changes encountered in the band power values of EEG signal bands after doing an exercise [25]. This hypothesis was proven by variations that occurred with alpha and beta frequency band power that investigated after implementing a maximal effort exercise and shows an increment in beta absolute power in a group of electrodes [26]. In our study, the best scoring classification model was KNN with 98.4% accuracy with a ratio of training data and testing data 80 : 20, which was found to be a high scoring model in other studies, especially when applied against applications with a low-dimensional [27] feature vector of data [28]. The KNN was found to perform effectively to extract and classify feature vector for different facial movements and expressions measured by noninvasive EEG devices. The accuracy was around 98% driven by implementing segmentation to the complete signal waveform [29]. Even though classification could be applied using other EEG features like the average spectral centroid, average standard deviation, or average energy entropy, but still the power spectral density offers the highest accuracy with all classifiers and was found to score 100% with KNN when analyzing EEG signals from different human cognitive states employed to control brain computer interface (BCI) devices [30]. In contrast to our work which investigated the effect of a single bout of acute exercise, the effect of increasing running exercise intensities on spontaneous EEG was investigated by a study, which found that the overall spectrum power in EEG significantly increased in all frequency bands with increasing intensities of exercise, lactate level has increased, and even after a period of 15- to 30-minute recovery, lactate enzyme level has decreased but still significantly higher than baseline and discernible [31]. The subsequent decrease in spectrum power was seen in a subset of frequency bands in some cortical regions suggesting a decrease in cortical activation after exercise intensities, as a hypothesis of brainstem inhibitory mechanism, may occur [32].  Table 4 shows the results of various objective studies comparable to our work.

The article "Classification of Lactate Level Using Resting-State EEG Measurements" was retracted in 2023. Reasons: signs of a paper mill; suspected computer-generated content; unreliable results or conclusions; lack of ethics approval or compliance.

## 5. Conclusions

The proposed work represents the use of band power spectral density along with machine learning techniques for classification and analysis of EEG signals recorded during resting-state tasks. The band's power feature of EEG signals was extracted using FFT for all of the 16 channels of each subject's EEG recording. Three different classification models (KNN, decision tree, and logistic regression) were applied, and their performance was reported. The classification accuracy of KNN and decision tree found to be above 98%. This makes the study the unique and pioneer one to discuss and prove the ability to use resting-state EEG signals as an accurate measure for the human tiredness level through predicting lactate enzyme level high or low. The band power was found to be a very useful EEG feature to classify these signals after performing acute exercise sessions. Hence, the proposed feature extraction and classification system have the significance to be applied on real-time EEG applications like BCI, IoT, military, or medical applications to predict the individual physical tiredness state that can assist in many crucial situations. As a suggested study expansion, the classifiers could be applied to EEG data collected for each subject individually with applying the same previous procedures, and the results could be compared in both cases. This may be implemented in future work possibly with applying more algorithms and preprocessing techniques for the purpose of achieving higher classification accuracy scores.

The article "Classification of Lactate Level Using Resting-State EEG Measurements" was retracted in 2023. Reasons: signs of a paper mill; suspected computer-generated content; unreliable results or conclusions; lack of ethics approval or compliance.

## Figures and Tables

**Figure 1:** The proposed classification model.

**Figure 2:** Cap 16-electrodes layout.

**Figure 3:** Pre and post exercise 16-channel EEG data.

**Table 1:** Classification score of applied models.

Model	KNN	Decision tree	Logistic regression
Accuracy	98.4%	98.0%	70.0%

**Table 2:** Sensitivity and specificity of the classifiers.

Model	KNN	Decision tree	Logistic regression
Sensitivity	98.8%	97.2%	76.5%
Specificity	97.0%	94.2%	64.0%

**Table:** (a) Precision values for decision tree

	Total	3867	3893	7760
Actual class	Lactate-level-low	3790	76	3866
	Lactate-level-high	77	3817	3894
		Lactate-level-low	Lactate-level-high	Total
		Predicted class		

**Table:** (b) Precision values for KNN

	Total	3870	3890	7760
Actual class	Lactate-level-low	3804	62	3866
	Lactate-level-high	66	3828	3894
		Lactate-level-low	Lactate-level-high	Total
		Predicted class		

**Table:** (c) Precision values for logistic regression

	Total	4359	3401	7760
Actual class	Lactate-level-low	2959	907	3866
	Lactate-level-high	1400	2494	3894
		Lactate-level-low	Lactate-level-high	Total
		Predicted class		

**Table 4:** Score results of various objective studies.

Study	Year	Electrode no.	Study objective	Applied algorithms	Accuracy %
[29]	2016	14	Classify facial movement and expressions by a noninvasive EEG signals	KNN	98.0
[30]	2018	1	Analyze EEG signals from different cognitive states to control BCI devices	LDA, SVM, KNN	95.0, 100.0, 100.0
[33]	2014	128	EEG signal classification recorded while doing a complex cognitive task	ANN, SVM, MLP, KNN, Naïve Bayes	88.89, 98.75 98.57, 98.21 83.57
[34]	2016	12	Monitoring EEG signal while driving to detect the driver fatigue state	SVM	91.28
[35]	2019	19	EEG signal features extraction and classification during fatigue exercise	SVM	90.0
Present study	2020	16	Classify resting-state EEG to predict lactate, high or low	KNN, DT, LR	98.4, 98.0, 70.0

## Data Availability

The EEG dataset which was used in the present study is available from the author, Adil Deniz Duru, through a reasonable request.
